The article "Design of Interactive Vocal Guidance and Artistic Psychological Intervention System Based on Emotion Recognition" was retracted in 2023. Reasons: signs of a paper mill; suspected computer-generated content; unreliable results or conclusions; concerns about the data.

# Design of Interactive Vocal Guidance and Artistic Psychological Intervention System Based on Emotion Recognition

**DOI:** 10.1155/2022/1079097

**Published:** 2022-06-17

**Authors:** Wenwen Mo, Yuan Yuan

**Affiliations:** ^1^Human Resources Office, Sichuan College of Traditional Chinese Medicine, Mianyang, Sichuan 621000, China; ^2^School of Marxism, Northwestern Polytechnical University, Xi'an, Shaanxi 710072, China

## Abstract

The research on artistic psychological intervention to judge emotional fluctuations by extracting emotional features from interactive vocal signals has become a research topic with great potential for development. Based on the interactive vocal music instruction theory of emotion recognition, this paper studies the design of artistic psychological intervention system. This paper uses the vocal music emotion recognition algorithm to first train the interactive recognition network, in which the input is a row vector composed of different vocal music characteristics, and finally recognizes the vocal music of different emotional categories, which solves the problem of low data coupling in the artistic psychological intervention system. Among them, the vocal music emotion recognition experiment based on the interactive recognition network is mainly carried out from six aspects: the number of iterative training, the vocal music instruction rate, the number of emotion recognition signal nodes in the artistic psychological intervention layer, the number of sample sets, different feature combinations, and the number of emotion types. The input data of the system is a training class learning video, and actions and expressions need to be recognized before scoring. In the simulation process, before the completion of the sample indicators is unbalanced, the R language statistical analysis tool is used to balance the existing unbalanced data based on the artificial data synthesis method, and 279 uniformly classified samples are obtained. The 279∗7 dataset was used for statistical identification of the participants. The experimental results show that under the guidance of four different interactive vocal music, the vocal emotion recognition rate is between 65.85%-91.00%, which promotes the intervention of music therapy on artistic psychological intervention.

## 1. Introduction

With its harmless, simple, and relaxing characteristics, music therapy has become an important means of alleviating artistic psychological intervention that has been gradually paid attention by people [1–3]. The so-called music therapy is to make the performer inject emotion into the music through the corresponding relationship between music and emotion and guide the performer's emotion through communication and counseling, so as to correct the cognition and relieve the performer's existence. The problem of artistic psychological intervention is to give full play to the therapeutic function of music. The important value of the existence of higher art colleges is to cultivate more artists and performers. If many outstanding students give up the stage and ideals because of the psychological intervention of art, this will not only affect their own development but also affect the school and society. At present, the form of music therapy is gradually being valued by people. As a new type of therapy, music therapy takes the function of music as the basis and intervenes the performers through various forms of music, so as to relieve the performers' artistic psychological intervention. This paper studies and analyzes the psychological intervention of music therapy in vocal music performance students' artistic psychological intervention [4–6].

In response to the above situation, various countries have invested a lot of energy to carry out related research. For example, the affective computing group of a laboratory in the United States is specialized in how the computer samples the signals in the surrounding environment and how the computer makes the collected signals [7–9]. Zhang et al. [10] believe that the signals sampled by the computer include physiological signals of the human body signals and vocal signals. Hasnul et al. [11] analyzed the characteristics of different emotions in the vocal music signal, then obtained the relevant emotional characteristics, and finally judged what kind of state the signal to be tested expresses. Considering that the number of high-risk feature words in the real text is relatively small, the more common ones are still the words with average risk level, and the frequent occurrence of feature words with average risk level will greatly increase the risk of the text. The above is the content of vocal music emotion recognition. Lima et al. [12] analyzed that sound is often used by humans to express inner feelings and is one of the ways of communication. Geraets et al. [13] believe that the emotional information contained in the signal becomes an important channel for understanding things.

This paper uses self-made questionnaires to understand the psychological intervention status of the subject's art and uses self-made therapeutic music to intervene on the subject's nervousness, correcting his cognition, changing his behavior, alleviating and eliminating the subject's artistic psychological intervention, and improving the overall mental health of the students. The vocal emotion recognition algorithm based on convolutional neural network is studied. Firstly, the convolutional neural network is trained, in which the feature input is a matrix composed of emotional features of Mel-frequency cepstral coefficients, and finally, the vocal music of different emotional categories is recognized. The vocal music emotion recognition experiment based on convolutional neural network is carried out from the two aspects of emotion type and the number of training sets. The experimental results show that the intersection idea and smote artificial data synthesis method are used to preprocess the data, eliminate the invalid data and balance the unbalanced data. Finally, 279 samples and 76 indicators were obtained (including homework scores, video viewing rate, courseware access times, the number of exchange posts in the discussion area, the proportion of vocal music guidance in the chapter, and artistic psychological intervention test scores). Subsequently, the Lasso regression algorithm was used to screen 76 indicators and the remaining 7 network participants' vocal music guidance behavior indicators (vocal guidance chapters, vocal guidance duration, number of posts in the discussion board, homework 1, homework 3, homework 4, and video viewing ratio) to participate in the subsequent model establishment. At the same time, the index screening of the Lasso regression algorithm effectively reduces the kappa value between the indexes from 1.3018 to 2.7768, which effectively avoids the multicollinearity problem of the model.

## 2. Methods

### 2.1. Emotion Recognition Signal Solution

In the research on facial emotion recognition expressions, the viewpoints that there are five different emotions including happiness, fear, sadness, anger, and disgust have been recognized and adopted by more researchers [14, 15]. It can be seen that the number of instances between classes is extremely unbalanced, and the IR ratio between the minority class and the majority class is very different. From experience, class imbalance will have an impact on the accuracy of the detector. The effect of foreground-foreground class imbalance should be taken into account in object behavior detection [16–19].

(1) $$\begin{array}{c} y\left(i,j\right)=1-\cos\left(i\times pi-a\right)-\sin\left(j\times pi-b\right)-c. \end{array}$$

Adding a feature fusion network to the detection model will increase the complexity of the model to a certain extent, but this complexity has little impact on the detection model. Because emotion recognition only does 4 1 × 1 convolutions, 4 upsampling, and 4 addition operations in the feature extraction network, this method allows the detection model to perform emotion recognition on multiple scales, making the detection model, and the classification accuracy has increased significantly. The complexity brought by emotion recognition to the detection model is relative to the improvement of classification performance, and the impact of this complexity is completely acceptable.

Due to the relationship between the feature points, the input data can be regarded as a series of features with time information on a fixed graph, so the graph-based identification method is mainly selected. The width of the main lobe of the rectangular window is smaller, and the peak value of the side lobe is larger, and the resolution of the frequency spectrum is higher, so its frequency spectrum leakage phenomenon is more serious, while the side lobe width of the Hamming window is lower and the side lobe attenuation is more serious, with good low-pass characteristics. If the purpose is to reflect the frequency spectrum characteristics of short-term vocal signals, compared with the two types of window functions, the Hamming window is more suitable [20–25].

(2) $$\begin{array}{c} f\left(m,n\right)=\left\{\begin{array}{cc} \frac{1}{\left(m+n\right)/\left(m-n\right)}, & 0<n<m<1,\\ 0, & \text{otherwise}. \end{array}\right. \end{array}$$

To conduct mining and analysis of network performance data, first perform data preprocessing and delete useless indicators: the index values are exactly the same, that is, useless; delete duplicate indicators: the index values show the same performance, but the index names are different; delete nonvocal guidance behavior indicators: each time for the performance index of the artistic psychological intervention test is deleted, because the final score of the subject is weighted by the results of the artistic psychological intervention test of the class. Data balance processing: since the final score of the subject is seriously unbalanced, which affects the generalization ability of the model, the SMOTE algorithm is used, carrying out data balance processing; secondly, use Lasso algorithm to filter the remaining indicators. Finally, the XGBoost model is established with the above 7 object vocal guidance behavior indicators.

### 2.2. Interactive Vocal Guidance Mechanism

After the vocal signal is framed, a new vocal sequence will be generated, and this new vocal sequence will change with time. After the framing operation, the characteristics of the vocal signal can be described more conveniently and accurately. The vocal signal can be processed to be short-term stable during analysis, but in real life, the speaker's speech is not always intermittent. If the overlap between adjacent subframes is adopted, the overlapping part is called frame shift. If the overlapping method is used in the analysis, the vocal signal after the framing operation will be able to express the original vocal signal well, generally taking about 33 to 100 frames per second.

(3) $$\begin{array}{c} h\left(x,y\right)=1-{ax}^{\left(i,1\right)}-{by}^{2\left(i,2\right)}-c. \end{array}$$

Annotate all visible objects with class labels and bounding boxes on every frame in the clip. The VID dataset has a total of 30 categories, and the dataset consists of three parts: training set, validation set, and test set. The training, validation, and test sets in the initial version of the VID dataset contain 1952, 281, and 458 segments, respectively. The feature map of the vocal signal is obtained through the feature extraction network, and then, the feature map is input into the RPN network, and the candidate region (proposal) is generated on the feature map, and a part of the candidate region is selected according to certain rules, and the candidate region is obtained by combining the feature map through the ROI pooling operation.

For the vocal music instructors collected in Figure 1, the ten tables contain not all the same personnel information. In order to obtain more and comprehensive index information, this paper uses the idea of intersection to select the data of 149 famous vocal music instructors from all vocal music coaching behavior tables, including a total of 90 indicators. Among the 90 indicators, there are 11 indicators with the same value but different names and 3 indicators with the same value. Delete the above indicators, and finally, there are 149 rows and 76 columns of data. Among them, homework 1 to homework 9 represent the scores of the first to the ninth homework. The ratio of random events and probability learning represents the proportion of vocal music instruction in Chapter 1 and curriculum development overview and the three elements of probability. The proportion of vocal music instruction represents the first chapter.

### 2.3. Intervention System Frequency Resonance

The usual framing method of vocal intervention system can be understood as follows. The final completion of the framing step of the vocal signal is completed by applying a window function. The length of the window function is limited. Specifically, the window function *w* and the amplitude value of the vocal signal sample are set to zero, and the currently required vocal subframe is obtained at this time. An area under the ROC curve of 0.5-0.7 indicates a low diagnostic value; 0.7-0.9 indicates a moderate diagnostic value; and above 0.9 indicates a high diagnostic value. The areas under the four ROC curves in this study are all between 0.7 and 0.9, indicating that the diagnostic value of this research method is moderate, and it can be used to identify and diagnose the risk of text.

(4) $$\begin{array}{c} s\left(m,n\right)=\frac{ds\left(m\right)}{ds\left(n\right)}-\frac{d^{2}s\left(m\right)}{{ds}^{2}\left(n\right)}-\cdots -\frac{ds\left(m-i\right)}{ds\left(n-j\right)}. \end{array}$$

The SMOTE algorithm is mainly aimed at balancing unbalanced data, which is an extremely critical step in the research process of this paper. The Lasso regression algorithm is used to screen model indicators, and at the same time, it can reduce the multicollinearity problem of the model, so that the indicators used in the model are within a reasonable range, and the selected indicators can be applied to the model. The XGBoost model is integrated and developed on the basis of the tree model, and its high efficiency, fast speed, and strong stability have laid a solid theoretical foundation for the research work of this paper. According to the quality of the model effect, this paper uses the precision rate, recall rate, and *F* value to discuss. The precision rate and the recall rate contradict each other to a certain extent, so the *F* value is introduced (the *F* value is the weighted average of the precision rate and the recall rate). According to the different weight settings of the precision rate and the recall rate, there are *F*1 value and *F*2 value. The *F*1 value is mainly used in this study.

After the data in Table 1 is balanced, the dimension of the data analyzed in this paper is 279 × 76, but since the final score of the subject is obtained by adding the weights of the midterm artistic psychological intervention test, the final artistic psychological intervention test, and the usual test, therefore, the artistic psychological intervention of the correlation coefficient between the tested metric and the subject's final score is too large. Moreover, the purpose of this paper is to explore the relationship between object network behavior and its final vocal music instruction course score, so 4 indicators of artistic psychological intervention test are artificially discarded. In addition, there are many homogeneous indicators. In this paper, kappa analysis method is used to conduct multicollinearity analysis on the existing indicators, and *K* = 1.301819e + 18, which is far greater than 1000. Therefore, indicator screening becomes necessary.

## 3. Results

### 3.1. Statistics of Artistic Psychological Data

Through the statistics of the survey data of the artistic psychological questionnaire, it can be seen that among the 80 valid questionnaires, there are 10 subjects with severe artistic psychological intervention, accounting for 12.5% of the effective test population. There are 23 subjects with “anxiety,” accounting for 28.7% of the effective test population; 27 subjects with mild artistic psychological intervention, accounting for 33.7% of the effective test subjects; 20 subjects without artistic psychological intervention; and 25% of the number of valid tests. From the survey data, it can be seen that among the subjects of vocal music performance, the problem of artistic psychological intervention is relatively common.

(5) $$\begin{array}{c} \left(\begin{array}{cc} \Delta d\left(1,1\right) & -1\\ 1 & \Delta d\left(1,1\right) \end{array}\right)=\left(\begin{array}{cc} \frac{ds\left(m\right)}{ds\left(m\right)} & 0\\ 0 & \frac{ds\left(n\right)}{ds\left(n\right)} \end{array}\right). \end{array}$$

The first use of this hierarchy was for SSDs. But feature maps of different depths will lead to different amounts of semantic information. High-resolution feature maps mainly contain low-level feature representations, and these low-level features can impair the representational ability when recognizing objects. In order to avoid using low-level features, SSD builds feature pyramids from the high-order bits of the feature extraction network to achieve object detection at different scales. As we all know, the low-level features contain less semantic information, but more target location information, and the high-level features contain rich semantic information, but the target location information is very rough. As a result, this attempt at SSD misses the opportunity to use low-level features that are very important for detecting small objects.

(6) $$\begin{array}{c} \text{termeal}\left(org\left(i,j\right),i,j\right)=\overset{n-1}{\underset{i=0}{\sum }}\frac{t_{i}\left(i,j\right)*s_{i}\left(i,j\right)-org\left(i,j\right)}{i-j}-\frac{esc\left(i^{\prime },j^{\prime }\right)}{ds\left(i\right)/ds\left(j\right)}. \end{array}$$

After SPSS reliability analysis, the overall Pearson correlation coefficient of the questionnaire was calculated, and its internal consistency reliability was above 0.9. Compared with the survey results of the classic questionnaire (2), the results of emotion recognition screening were equivalent, indicating the compiled emotion recognition. The scale has good validity. The number of instances in the “raise hand” category is more than that of “standing” and “turning around,” but the AP is not as high as these two; even when the IOU values are 0.50 and 0.10, the situation is the same. The diversity is much more than standing and turning.

Then, by comparing the index of the weighted risk score calculated by using the basic thesaurus of risk text features and the expanded thesaurus, respectively, it is found that the index of the weighted risk score calculated by using the basic thesaurus of risk text features is higher (0.648 > 0.614), indicating that this method is relatively optimal for risk text recognition. When the diversity of a category is higher, the number of instances should be relatively larger. Moreover, the questionnaire has the following characteristics compared with the questionnaire; the content of its detection is mainly the characteristic aspect of emotion recognition, that is, which people are usually more likely to have emotion recognition, rather than just measuring the severity of a certain emotion recognition. From the point of view of score significance, it is more meaningful to measure trait anxiety and identify objects that are usually easily affected by performance anxiety than to measure state emotion recognition, and some targeted prevention and intervention can be done in advance.

### 3.2. Special Classification of Emotion Recognition

The artistic psychological signal biofeedback therapy instrument is used to measure physiological indicators such as heart rate, breathing test, and artistic psychological signal for the emotion recognition of the two groups. The test data includes the following four stages: start test, breathing relaxation stage test, and music therapy stage test. In the recovery stage test, the effect of therapeutic music on alleviating the psychological intervention of art was analyzed through the statistics of the subjects' heart rate, respiratory rate, and psychological signals of art and other physiological indicators, after computer processing and comparison.

(7) $$\begin{array}{c} t\left(m\right)-t\left(n-m\right)\frac{t_{i}\left(m\right)\cdot s_{i}\left(m\right)-u\left(n,m\right)}{n-m}=\text{escaper}\left(m^{\prime },n^{\prime }\right). \end{array}$$

In the process of listening to the therapeutic music, the artistic psychological signal values in all test stages changed, among which the artistic psychological signal value in the initial testing stage was low, while the value in the breathing test stage was the highest. The recovery test phase is gradually flattened. Because the accumulated loss will be relatively large, most emotion recognition algorithms increase the penalty cost of misclassification of small categories from a cost-sensitive point of view and directly reflect this cost in the objective function. The foreground-background imbalance problem is generated during training and has nothing to do with the number of instances in Figure 2, and its imbalance ratio is often much higher than that between foreground-foreground categories.

A total of 61 subjects participated in this experiment, and the subjects were surveyed and given feedback before and after the experiment. Overall, in this intervention test, the subjects of vocal music performance have achieved the purpose of adjusting heart rate and strengthening breathing depth and greatly improved the psychological intervention of art; the subjects' body circulation is accelerated and can maintain a state of relaxation, thus confirming the function and effect of music therapy on alleviating the psychological intervention of art. In addition, it can also be found that when the positioning accuracy of the prediction frame is higher, that is, when the IOU value is 0.75, the AP of the “head-up” category is still the highest among all categories, at 75.6%, which is far higher. For several other categories, this shows that the number of category instances in the training set is sufficient to ensure the accuracy of its classification. When the IOU value is 0.75, the classification AP of the “raise hand” category is the lowest among the six main categories, with an AP of only 19.6%.

### 3.3. Interactive Vocal Guidance Coding

The frequency range of vocal signals is usually 300 to 3400 Hz. Since the average power spectrum of the vocal signal is affected by the glottal excitation and the radiation from the mouth and nose, the high-frequency end drops by 6 dB/octave above 800 Hz, so when finding the spectrum of the vocal signal, the higher the frequency, the smaller the corresponding component, so do preemphasis in the preprocessing. The purpose of pre-emphasis is to enhance the high-frequency part, smooth the spectrum of the signal, keep it in the whole frequency band from low frequency to high frequency, and use the same signal-to-noise ratio to obtain the spectrum, which is convenient for spectrum analysis or channel parameter analysis. The preprocessing step for the signal of Figure 3 is done using a first-order high pass filter.

And the evaluation methods of the two modules need to use the results of action recognition or expression recognition. After the solution of converting video data into feature points has been selected, it is necessary to consider how to perform action recognition and expression recognition based on the coordinates of feature points.

A total of 29 subjects participated in the experiment. We conducted psychological surveys and information feedback on the subjects before and after the test to assess whether their stress levels improved. In this intervention activity, therapeutic music has played a role in adjusting heart rate, strengthening breathing depth for both the group and the Bel Canto group, and showing that the therapeutic music can relieve and change the tension state; the artistic psychological signal response has returned to normal, showing an increase in skin current, the circulation is accelerated, the body is in a warm state, and the relaxation effect is achieved; it shows that the therapeutic music can effectively relieve the psychological intervention of the subject's art. According to the statistics of the feedback questionnaires filled out by the subjects, 87% of the subjects indicated that the therapeutic music has achieved the effect of alleviating the psychological intervention of art.

## 4. Discussion

### 4.1. Emotion Recognition Signal Extraction

The cepstrum separates the fundamental harmonic of emotion recognition from the spectral envelope of the vocal tract. The low-frequency part of the cepstrum can analyze the vocal tract, glottal, and radiation information, and the high-frequency part can be used to analyze the excitation source information. The periodic excitation of the voiced signal is reflected in the cepstrum as the impulse of the same period, so the pitch period can be estimated from the cepstrum waveform. Generally, the second impulse in the cepstral waveform is regarded as the fundamental frequency of the corresponding excitation source. If the peak of the cepstrum exceeds the set threshold, the input vocal segment is classified as voiced, and the position of the peak is an estimate of the pitch period. If the threshold peak is not exceeded, the input vocal section is unvoiced. In the experimental process of expression recognition, it was found that the random forest has a high classification accuracy for the feature point sequence in the unit of pictures, so the random forest was determined as the main classifier for expression recognition, and the expression intensity and pleasure were analyzed. After the relationship with the expression category, the scoring method is designed.

On the basis, two scales are added, and the feature maps of each convolutional layer are fully utilized to obtain features of different scales. The path of feature fusion is from top to bottom, upsampling the feature map of each scale from top to bottom with a step size of 2, and performs a 1 × 1 convolution operation on the original feature output of the convolution layer to achieve horizontal connection. The graph is added, and the feature size of the adjacent feature layers is doubled, and the object behavior detection is performed on these five feature levels with different scales. According to the principle of music heterogeneity and isomorphism, it induces and regulates the synchronous resonance of emotions and guides the subjects to change from emotion to behavior; the music rhythm is soothing, steady, and light, which is consistent with the breathing rhythm of the human body, so that people can relax and decompress as soon as possible. The nonsemantic function of music helped the subjects to open the door of the subconscious, so that the mind could be deeply channeled and relaxed.

(8) $$\begin{array}{c} t\left(m\right)-t\left(n-m\right)=\left\{\begin{array}{cc} t\left(m\right)+t\left(n\right), & m>n,\\ \frac{-\left(m-n\right)}{t\left(m\right)+t\left(n\right)}, & m<n. \end{array}\right. \end{array}$$

If we set the threshold to 0.48, the model has the highest accuracy on the 1st dataset. The accuracy rate is equal to 0.54, which means that 46% of the data are misclassified as positive, the recall rate equal to 1 means that no samples are misclassified as negative, and the *F* value is 0.35, which means that the overall accuracy of the model is not very high, and there is still a lot of room for improvement. At the same time, the training results of the model are predicted ten times, only the second prediction accuracy rate is 96, and the prediction accuracy rate of the other models is 100%. The average prediction accuracy of the model trained ten times is 99.6%.

### 4.2. Aggregation of Interactive Vocal Guidance Elements

Interactive music is a regular wave shock, which is transmitted into the body through the human auditory organs and auditory nervous system, causing the body cavity to generate regular resonance, so that the body movement is in a harmonious and orderly state; music sound waves stimulate the central nervous system, make the endocrine system produce hormones that are beneficial to the body and mind, and promote the body's metabolic function; music can distract attention and affect the function of the brain and can appropriately relieve physical pain. The specific experimental parameter configuration for training and testing is shown in the text, and the name, value, and interpretation table of each parameter are described in the table. Among them, during training, the classification loss function and box regression loss function in the rcnn stage are *i*, respectively, and the hyperparameters during training.

The feature map of the first scale is upsampled with a step size of 2, and the original feature map of the previous scale is subjected to a convolution operation with a psychological signal node size of 1 × 1 and a psychological signal node number of 256. The feature map is added to obtain the feature map of the second scale (scale-2). According to the same fusion method, the feature maps of the third scale (scale-3), the fourth scale (scale-4), and the fifth scale (scale-5) can be obtained. The red-dotted box in the figure represents the feature fusion algorithm as described above. It shows that the average scores of both male and female subjects are higher than the norm in anxiety and nervousness. At the same time, it is not enough to judge the start of a person's action from the distance or the direction change alone. In the performance of children with autism, there may be a start action that changes the distance, but the direction does not change (when the action starts, the hand is raised upward, the distance change is the most obvious, and the angle change is smaller). From the perspective of personality factors, the subjects were more prone to nervousness and anxiety.

### 4.3. Simulation Realization of Artistic Mental Model

The data acquisition, recording, and analysis system of the artistic physiological coherence and autonomous balance system (SPCS) was used to connect the computer for recording and analysis; at the same time, the VIEWSONIC computer audio player was used to play the experimental music to the subjects through headphones. The method of extracting formants in this paper adopts the cepstrum method. The cepstrum separates the fundamental harmonic and the spectral envelope of the vocal tract. The low-frequency part of the cepstrum can analyze the vocal tract, glottal, and radiation information, while the high-frequency part can be used to analyze the incentive source information. The low-frequency window selection is performed on the cepstrum, and the output after DFT is the smoothed logarithmic modulus function. This smoothed logarithmic spectrum shows the resonance structure of a specific input vocal segment; that is, the peak of the spectrum basically corresponds to the formant frequency. By locating the peaks in the smoothed log spectrum, the formants can be estimated.

In the process of listening to the music, the subjects' artistic psychological signal values have obvious changes. The artistic psychological signal index in the baseline stage is low, and the artistic psychological signal index shows an upward trend in the breathing stage and tends to be flat in the meditation stage and recovery stage, reaching normal. Index. When the threshold in Figure 4 is 0.10 (that is, when the positioning error is ignored), the Loc value is 71.9%. Compared with C50, the AP is only increased by 2.9 percentage points, which means that when the IOU value is 0.50, the prediction frame roughly surrounds the target object. After removing the confusion of different categories, the value of *i*-th is 88.9%. Compared with Loc, the AP is increased by 17 percentage points (the green area in the figure), which means that the prediction frame surrounds the object, but a large proportion of the objects are classified incorrectly. After removing the false positives on the background, the value of BG is 90.7%. Compared with *i*-th, the AP is only improved by 1.8 percentage points, which means that most of the areas enclosed by the prediction frame are positive samples (not the background area).

The subjects' breathing ratio was shallowest during the baseline period. With the intervention of therapeutic music, the breathing depth index of the subjects in the breathing phase gradually increased and reached the best state. This is because the subjects were fully relaxed by doing muscle relaxation and breathing training under the guidance of background music and introduction. It begins to decline during the meditation phase and begins to increase in depth from the recovery phase.

### 4.4. Example Application and Analysis

When aiming at different emotion recognition tasks, due to the different requirements for the positioning accuracy of the target frame, whether to use mAP as the model evaluation standard can be determined according to the specific situation. In this paper, the localization of the object does not need to be very accurate, so AP is not used as the evaluation criterion. The ROC curve does not perform as well as the PR curve in the case of extremely class imbalanced classification and informed to keep the body posture as much as possible during the test and not to move freely. During the experiment, the subjects closed their eyes and lay flat on the bed in the music psychology laboratory naturally, connected the signal detector of the SPCS system to the designated position of the subjects, and played therapeutic music to the subjects. Therefore, in this project, the Euclidean distance and the cosine angle are calculated, respectively, and the minimum value is taken after the starting frame is obtained. For individual training classes that expect explicit action feedback, this calculable change can reflect the speed of students' response to task instructions and the level of student engagement in the current class.

The left form of the addition represents the cepstrum of the excitation sequence, and the right form of the addition refers to the cepstrum of the channel impulse response. Experimental results show that the phenomenon of fast decay occurs in the cepstrum of the vocal tract response. Therefore, it is necessary to build a cepstral filter, which has the function of cepstral separation of analog channels. In order to reduce the interference of glottal excitation, it is necessary to add an inverse filter in the cepstral domain. In the baseline stage, the breathing rate of the subjects was relatively unstable. When the therapeutic music began to intervene, the breathing frequency of the subjects in the breathing stage began to stabilize and showed an upward trend. In the meditation stage, it returned to a more normal state, and the state began to rise in the recovery stage.

In the emotion recognition task, when evaluating the accuracy of classification, the evaluation in Figure 5 is usually combined with the accuracy of the positioning of the prediction frame. The evaluation standard for measuring the positioning accuracy of the prediction frame is IOU, which represents the intersection ratio of the target frame and the prediction frame. The positioning accuracy of the detection frame is very high, as long as the prediction frame can roughly surround the object. In this paper, when evaluating the accuracy of the classification, the IOU value is 0.5. Based on the above experience and practice, the network prediction performance of the number of emotion recognition signal nodes in different artistic psychological intervention layers is compared by trying methods, and the number of emotion recognition signal nodes with relatively good recognition results is selected as the number of emotion recognition signal nodes in the artistic psychological intervention layer. In the experiment, the number of emotion recognition signal nodes in the artistic psychological intervention layer ranges from 10 to 35.

## 5. Conclusion

After emotional recognition of the interactive vocal guidance module, the artistic psychological intervention system scoring module finally outputs the participation score, and the expression scoring module finally outputs the expression pleasure score and expression intensity score. These three scores are all related to the artistic psychological intervention object and performance. Subsequently, related psychological intervention studies on online vocal music coaching have shown that multimedia technology, peer feedback, cooperative vocal music coaching, simulation games, and even mandatory constraints on the subject's vocal music coaching behavior can effectively reduce the mind wandering and focus of online vocal music coaches. In the end, it will improve the efficiency of its vocal music guidance and ensure the effective implementation of online courses. The core of the project can be divided into two parts, the first part is action recognition and expression recognition, and the second part is the evaluation method based on its results. Through experiments, it has been proved that emotion is positively correlated with participation, and the emotional pleasure score and expression intensity score are also positively correlated, so the performance of artistic psychological intervention objects should be the same as participation score, expression pleasure score, and expression intensity. The scores are all positively correlated. When there is no data to prove that the importance of the three scores to the final score is different, the weights are considered to be 1, so the final evaluation of the performance of artistic psychological intervention objects can be achieved. The kappa value also changed from 1.3018 to 2.7768, avoiding multicollinearity effects among variables. Under the tenfold cross-validation, the XGBoost algorithm was used to predict the results of 279 subjects, and the average prediction accuracy reached 99.6%. In the intervention of the online object's vocal music instruction process, the instructor's sense of participation is too low, and the online vocal music instructor's vocal music instruction process can be added to guide the object to approach the discussion area and improve the object's mutual feedback behavior.

## Figures and Tables

**Figure 1:** Topology of interactive vocal guidance mechanism.

**Figure 2:** Disproportionately specific classification of emotion recognition.

**Figure 3:** Coding distribution of interactive vocal guidance channel parameters.

**Figure 4:** Value distribution of artistic physiological coherent balance signal.

**Figure 5:** Prediction distribution of interactive vocal signals under emotion recognition.

**Table 1:** Description of frequency of psychological intervention system.

Intervention index	*F*1 value	*F*2 value	*F*3 value	*F*4 value
10	0.396	0.719	0.127	0.834
20	0.449	0.433	0.187	0.917
30	0.770	0.764	0.824	0.286
40	0.431	0.426	0.490	0.461
50	0.113	0.881	0.186	0.674
60	0.121	0.993	0.322	0.380

## Data Availability

The data used to support the findings of this study are available from the corresponding author upon request.
